RETRACTED

# SFN: A Novel Scalable Feature Network for Vulnerability Representation of Open-Source Codes

**DOI:** 10.1155/2022/2998448

**Published:** 2022-08-12

**Authors:** Junjun Guo, Zhengyuan Wang, Li Zhang, Yang Xue, Kai Long, Xin Jing, Jing Cheng, Guiping Li

**Affiliations:** School of Computer Science and Engineering, Xi'an Technological University, Xi'an, Shaanxi, China

## Abstract

Vulnerability detection technology has become a hotspot in the field of software security, and most of the current methods do not have a complete consideration during code characterizing, which leads to problems such as information loss. Therefore, this paper proposes one class of Scalable Feature Network (SFN), a composite feature extraction method based on Continuous Bag of Words and Convolutional Neural Network. In addition, to characterize the source code more comprehensively, we construct multiscale code metrics in terms of semantic-, line-, and function granularity. In order to verify the effectiveness of the SFN, this paper builds a Scalable Vulnerability Detection Model (SVDM) by combining SFN with Bi-LSTM. The experimental results show that the proposed SVDM can obtain precision over 84.3% and recall at 83.4%, respectively, while both FNR and FPR are less than 17%.

## 1. Introduction

Vulnerability is one of the main factors leading to software security problems, and vulnerability detection is an important means of discovering the existence of security problems in software. Due to the high complexity of software and the exploitability of vulnerability, the existence of vulnerabilities is almost inevitable [1].

At present, researchers have carried out a lot of work, and the source code-based vulnerability detection methods are mainly divided into dynamic analysis and static analysis. Dynamic analysis is to check the program status on the basis of execution. Common techniques include fuzzing and symbolic execution. The accuracy of dynamic analysis is relatively high, but there is a limitation that it is not easy to find the analysis spot, and there are problems such as low code coverage and missed reports, so dynamic analysis is subject to large limitations [2].

Static analysis is to find the vulnerabilities in the code by lexical, syntactic, and semantic analysis of the program to be tested without running the program [3]. According to the analysis object, static analysis mainly includes source code and binary analysis. Binary vulnerability analysis and mining methods can directly analyze the vulnerabilities in the binary code, and the accuracy is relatively high, but the analysis is more difficult [4]. Because of the rich and relatively complete semantic information, the vulnerability analysis can take into account the executable path of the program, so it is preferred by many researchers. Source code vulnerability mining methods mainly include logic-based reasoning and intermediate representation-based method. Logical reasoning-based methods describe the source code formally and use mathematical reasoning, model detection, and theorem proving to determine whether there is a specific type of vulnerability in the program. The method based on logical reasoning is based on a mathematical derivation process, so the analysis is rigorous and accurate, but the derivation process is complex and not suitable for the analysis of large-scale software. The method based on intermediate representation is to translate the source code into intermediate results that are easy to analyze and at the same time perform lexical/syntactic analysis and data flow/control flow analysis on the source code as needed to determine whether the source program contains vulnerabilities.

RETRACTED

With the development of deep learning, researchers are trying to apply deep learning to the task of vulnerability detection. Unlike the fields of image processing or natural language processing, which have mature algorithms, deep learning-based vulnerability detection is not yet supported by very mature algorithms [5], and the introduction of network models from other fields is generally considered in vulnerability detection due to the large size of source code data, the complexity of the principles of vulnerability formation, the difficulty of extracting vulnerability features, and the low level of automation. In recent years, except for a few recent studies introducing deep learning models [6] commonly used in NLP and image processing fields such as Convolutional Neural Networks (CNN), Long Short-Term Memory (LSTM) networks, and Bidirectional Long Short-Term Memory (Bi-LSTM) networks, most studies use traditional machine learning models such as Support Vector Machines (SVM), Random Forest, and Parsimonious Bayes for vulnerability detection [7]. Therefore, improving and tuning on the basis of mature algorithms is a more appropriate way at present.

Considering that source code has the characteristics of language and the vectorized source code features can be extracted by a neural network with universal applicability, this paper proposes a Scalable Feature Network for vulnerability feature extraction and collects numerous source code files to build a scalable code metric data set. The data set is utilized on the proposed SFN to prove the superiority of the model's effectiveness.

### 1.1. Our Contribution

1. In order to characterize the source code more comprehensively, this paper characterizes the source code at three scales: semantic granularity metric, function granularity metric, and line granularity metric and constructs a multiscale code metric data set. By studying how to characterize the vulnerability source code at multiple granularities, we can make the sample contain as much information about the source code as possible, and the proposed method can better learn the vulnerability patterns and improve the detection results.
2. This paper proposes a Scalable Feature Network (SFN), which aims to extract features according to the different granularity of code metrics through a three-layer longitudinal feature extraction model constructed by CNNs and a Continuous Bag of Words (CBOW). Unlike other deep learning-based vulnerability detection methods, the feature extraction model proposed in this study reveals the implicit relationships between different metrics while preserving the code features, explaining the deeper semantic information of the code. And after the hierarchical feature extraction, the code features under different granularity are combined into a multidimensional feature vector by the feature fusion technique to provide the code features containing rich semantic information for the representation learning module in order to obtain a deeper representation and achieve higher detection accuracy and stronger robustness.
3. In this paper, we construct a Scalable Vulnerability Detection Model (SVDM) based on multiscale code metrics and SFN. Specifically, the semantic metrics are vectorized by CBOW and form multiscale code metrics together with function-level code metrics and line-level code metrics; CBOW and Convolutional Neural Network are applied as the core algorithms of the model to extract features from the multiscale code metrics, and the extracted features are considered as the input data of the classifier. Finally, the model is fine-tuned by parameters such as the number of hidden layers, learning rate, and iteration, and the model structure and parameter configuration with the best effect are selected according to the experimental results.

RETRACTED

### 1.2. Paper Organization

Section 2 introduces the overview of the proposed method and the specific details.  Section 3 describes the experimental setup and evaluation metrics and analyzes the comparison with other tools and methods.  Section 4 presents the related works, and Section 5 concludes the paper.

## 2. Methodology

In this section, a vulnerability feature extraction method is proposed based on multiscale code metrics, which performs vulnerability source code feature extraction via the Scalable Feature Network (SFN) and uses the extracted features for vulnerability characterization learning to explore the vulnerability patterns and knowledge implied in the code metrics. Therefore, we firstly describe the framework of the SFN and secondly provide a specific description for the proposed method.

### 2.1. Data Set Construction

#### 2.1.1. Data Preprocessing

Since the existing data sets are not sufficient to effectively train and evaluate the proposed model, firstly this paper investigates several public vulnerability databases in academia and collects vulnerability codes. This information is usually stored in textual forms, such as the common vulnerability databases Common Vulnerabilities Exposures (CVE) [8], National Vulnerability Database (NVD) [9], and Software Assurance Reference Dataset (SARD) [10]. Each sample in the vulnerability database has a uniquely identified ID. Different vulnerability databases cover different kinds of information, but they basically include vulnerability description, danger level, release date, and source code, which provided a reliable basis for in-depth research on vulnerability detection. Finally, this paper collected a total of 67,845 vulnerability samples from the three public databases introduced in the previous paper, mainly including two vulnerability types, CWE-119 and CWE-399. After de-duplication and other operations, a database containing 61,638 vulnerability samples is obtained.

The collected vulnerability code data contain redundant information, such as semantically irrelevant comments, blank lines, and invalid code. In order to remove the redundant information, the code slicing technique is required. The code slicing technique is a source code classification method proposed by Mark Weiser in 1981. Code slicing is a method that extracts the core elements of a program from complex code, and the extraction of the elements is one of the key steps in constructing a multiscale code metric.

#### 2.1.2. Generating Multiscale Code Metric

Traditional code metrics characterize source code in terms of software engineering, code properties, and specifications; however, to perform vulnerability detection tasks through code metrics, traditional code metrics alone cannot fully characterize source code, so it also requires a kind of metric that can characterize source code in terms of semantics; moreover, there are metrics belonging to different granularities in traditional code metrics, which can be divided into function granularity and line granularity of code. Therefore, the three granularities of code characterization, semantic metrics, function granularity metrics, and line granularity metrics are described as multiscale code metrics.

The key step in data set construction is to construct multiscale code metrics from the collected source code data. According to our definition, multiscale code metrics are divided into semantic metrics, function granularity metrics, and line granularity metrics, and this subsection will focus on the details of multiscale code metric construction.

*(1) Semantic Metrics*. The extraction of semantic metrics mainly involves the construction of word vectors from slices of code in text form distributed through the CBOW in word2vec. In this subsection, a mathematical definition of the concepts involved in semantic metrics is given below.

RETRACTED

**Definition 1 .**

(semantically relevant). Given a piece of code *C* = {*c*_1_, *c*_2_,…, *c*_*n*_}, where *c*_i_ is code statement, *c*_i_ ∈ *C*. If the *j*th *v*_*i*,*j*_(1 ≤ *i*, *j* ≤ *n*) variable of the *i*th statement has a call relationship with other statements *c*_*o*_(1 ≤ *o* ≤ *n*), the statement *c*_*i*_ and the statement *c*_*o*_ are considered to be semantically related.

**Definition 2 .**

(code slicing). Given a code *C* = {*c*_1_, *c*_2_,…, *c*_*n*_}, where *c*_*i*_ is an utterance, *c*_*i*_ ∈ *C*. Let *V*_*i*_={*v*_*i*1_, *v*_*i*2_,…, *v*_*in*_} denote the set of semantically related variables in the utterance *c*_*i*_. Then, the code slice is an ordered subset *S* of the source code fragments extracted from *C* based on the set of semantically related variables *V*_*i*_, where *S* ∈ *C*, and each statement in *S* recursively depends on the semantically related variables of *V*_*i*_.

**Definition 3 .**

(semantic metrics). Given a code *C* = {*c*_1_, *c*_2_,…, *c*_*n*_} and a set *V*_*i*_ of semantically related variables, and each variable in *V*_*i*_ belongs to a statement *c*_*i*_ in the set *C* (1 ≤ *i* ≤ *n*). Let the set *M* = {{*m*_11_, *m*_12_,…, *m*_1*n*_}, {*m*_21_, *m*_22_,…, *m*_2*n*_},…, {*m*_*m*1_, *m*_*m*2_,…, *m*_*mn*_}} denote the set of ordered code subsets S trained by the word vector model to transform into vectors of the set of integer sequences and {*m*_*i*1_, *m*_*i*2_,…, *m*_*in*_} denote that the *i*th statement in *S* contains *n* linearly independent quantities in the vector space.

Based on the definition given previously, the final purpose of semantic metric extraction is to calculate the set *M*. Each sample of the processed code slice file is distinguished by a separator, the first line of each sample is the sample number and the file to which the sample code belongs and the CVE-ID; the second line that starts to the penultimate line is the semantically related code slice part; the “0” and “1” in the last line represent whether the sample contains a vulnerability.

*(2) Function Granularity Metrics*. The extraction of function and line-level code metrics is the same as the semantic metrics, which are computed from a data set of semantically relevant code slices collected and processed. The data used in this paper comes from NVD, CVE, and SARD, where the samples contained in NVD and CVE are from real-world open-source software code, and the samples in SARD are code slices that are artificially constructed by mimicking the pattern of vulnerable code with typical vulnerability patterns. Since code metrics can quantify code well, vulnerability-related features such as code size, coupling, and complexity can be used as input features for vulnerability detection models. This part focuses on the computation and extraction of function-level code metrics.

RETRACTED

The function granularity code metric describes the text, size, and complexity characteristics of the function, where the vulnerability is located, including program length, number of vulnerability submissions, cyclomatic complexity, and maintainability index. The details are shown in Table 1.

The code metrics that can be directly obtained statistically from this code slice are *N*_1_=26, *N*_2_=20, *η*_1_=7,  and *η*_2_=14, and the rest of the function-level code metrics can be calculated based on the *N*_1_, *N*_2_, *η*_1_,  and *η*_2_. The rest of the code metrics for this sample are shown in Table 2.

With the above steps, the function granularity code metric for the given code slice sample can be computed and extracted. In addition, to construct the multiscale code metric data set, it is necessary to calculate the line-granularity code metric, and the specific calculation and extraction process are described in the next subsection.

*(3) Line Granularity Metrics*. Line-level code metrics are code metrics associated with specific lines of code in a code slice, and they characterize the properties of the code itself from a code text perspective, such as the size of the code, the vocabulary it contains, and other attributes. Among them, all line-level code metrics can be obtained directly from the code slices, except for the program vocabulary *η*. The same code slice is given in Figure 2 as an example.

The line granularity code metric that can be counted and calculated from this code segment is shown in Table 3.

It is worth noting that the number of different operators (*η*_1_), the number of different operands (*η*_2_), the number of all operators (*N*_1_), and the number of all operands (*N*_2_) are the base values for calculating the function granularity code metric. Although the two levels of code metrics characterize different properties of the same code slice, they also reflect that there is a certain implicit relationship between different code metrics, and this implicit relationship between codes can be learned by the neural network through the subsequent training of the deep learning model, which can improve the vulnerability detection results.

RETRACTED

### 2.2. The Proposed Method

In the field of image detection, before the advent of feature pyramid networks, many networks utilized a convolutional layer with a single high-level feature for downsampling for target recognition and classification. Similar to image detection, the source code expresses different code features in different granularities.

The multiscale code metrics used in this paper are designed to represent different levels of source code characteristics by granularity. The semantic metric is to represent the semantic relationships in the source code context, the function granularity code metric is to characterize the complexity of the function where the vulnerability is located, etc., and the line granularity code metric is to represent the characteristics of the source code text such as size and vocabulary. This differentiated granularity characterizes the source code in a manner similar to that of FPN in image processing. The structure of SFN is shown in Figure 3.

The network structure has two distinct advantages.

1. Hierarchical structure SFN uses a three-tier structure for feature extraction corresponding to three different levels of code metrics. This vertical hierarchical structure not only enables a comprehensive extraction of the code features of the given samples but also allows for the addition of layers to supplement the feature information as needed in subsequent studies.
2. Different neural networks are selected for different attributes of the metrics. It can be seen that for semantic metrics, SFN chooses CBOW as the feature extraction network, whose effectiveness in the field of vulnerability detection has been proven by a large number of experiments by previous researchers; for function and line-level code metrics, CNN is chosen as the feature extraction network because there are certain implicit relationships between the attributes of these two levels of code metrics, and with the excellent local attention mechanism of CNN, it is able to extract the intrinsic relationship between each metric and protect the integrity of source code features.

Since the SFN feature extraction network uses a complex network structure with a combination of CBOW and CNN, the overall feature fusion process is similar to pyramid fusion in late fusion. Due to the high dimensionality and the difference in vector matrices size after the training and extraction, the three vectors need to be downscaled and shaped to one-dimensional before they are input into the detection module. The downscaled vectors also need to be stitched into multiscale feature vectors via concat.

RETRACTED

In summary, the specific steps of the method are described as follows:

1. Before starting the algorithm process, two counters *c*_0_ and *c*_1_ are set to count the number of samples outputting “0” and “1,” respectively. Define *N* as the total number of samples, then *N*=*c*_0_+*c*_1_, and the evaluation indicators *P*, *R*, FPR, FNR, and *F*_1_-measure of the detection results are also calculated by *c*_0_ and *c*_1_.
2. The multiscale code metric samples *S*={*M*, *F*, *L*} are divided according to semantic metric, function granularity, and line granularity, which are fed into SFN for feature extraction. Among them, the semantic metric is extracted using CBOW, and the function granularity and line granularity are extracted utilizing CNNs containing asymmetric convolutional kernels, respectively. The extracted features are *t*_1_, *t*_2_, *t*_3_, and *𝔻*_*t*_1__=*𝔻*_*t*_2__=*𝔻*_*t*_3__==1, where *𝔻*_*t*_i__ denotes the dimension of the feature vector *t*_i_.
3. The feature vectors *t*_1_, *t*_2_, and *t*_3_ cannot be studied directly, and they need to go through a feature fusion stage. In this paper, three feature vectors are stitched together using concat to obtain the global feature vector *T*=*f*_concat_(*t*_1_, *t*_2_, *t*_3_) for the detection samples. These vectors are provided as the inputs to the classification detector known as Bi-LSTM in this paper.

## 3. Experimental Results

In order to verify the effectiveness of the SFN, this paper combines SFN with Bi-LSTM network to construct a Scalable Vulnerability Detection Model (SVDM) for vulnerability detection. Firstly, this section introduces the experimental environment, then introduces the evaluation indicators for performance judgment, and introduces the specific parameter settings in the experiment. In the end, we analyze the experimental results.

### 3.1. Experiment Environment

The SVDM vulnerability detection model was developed under Linux in *Python*, and the model was based on the Keras framework. The detailed configuration parameters of hardware and software are shown in Table 4.

### 3.2. Evaluation Indicators

To evaluate the validity of the SVDM fairly and comprehensively, five general and well-known evaluation metrics are implemented in this paper: precision (*P*), recall (*R*), false-negative rate (FNR), false-positive rate (FPR), and *F*_1_-measure. The formulas are shown in Table 5.

### 3.3. Results Analysis

The multiscale code metric data set constructed in section II is utilized on the SVDM in this section, and the data set is divided on the same benchmark, where 80% of the data are used for training, and the rest of the data are used for detection. Meanwhile, this paper also selects the well-known vulnerability detection tools Flawfinder and RIPS, the statement code metric-based vulnerability detection methods VCCFinder, VPM, and VulExplore. To compare on the same benchmark, the above models are retrained based on the multiscale code metric data set in this paper while Flawfinder and RIPS can directly perform vulnerability detection without additional training.

RETRACTED

Firstly, the SVDM proposed in this paper was utilized on both sampled and unsampled data sets, considering the imbalance between positive and negative samples in the data set. The results are shown in Table 6.

As seen in Table 6, the unsampled data set leads to an unusually high FNR and FPR for the model. Since the number of negative samples is significantly larger than the number of positive samples, the unsampled data set leads to an increased imbalance in the data set, and this significant difference causes the negative samples to affect the convergence of the network model parameters, resulting in detection results that do not meet expectations. Therefore, in the later experiments, all models and methods are oversampled during the training process to provide a balanced data set.

As can be seen from Section 2.2, the samples in the multiscale code metric data set are mainly collected from the CWE-119 and CWE-399. In addition to certain differences in the semantic features of these two vulnerability types in code slicing, there are also certain differences in the sample distributions of their function and line-level code metrics, as shown in Figures 4 and 5, where each subgraph is the distribution of a code metric in its respective value range.

Clearly, there are significant differences in the sample distribution spaces of some metric attributes of CWE-119 and CWE-399. To verify the generalizability of the SVDM vulnerability detection model, the above two vulnerability types are tested here separately and in a mixture, using data from CWE-119-SET, CWE-399-SET, and the mixed data set of the two vulnerabilities, using Multi-SET, respectively. The detection results are shown in Table 7.

It can be seen that there are some differences in the training and detection results of the three data sets, where CWE-399-SET has better experimental results. This is because, firstly, the number of vulnerability samples from SARD in CWE-399 is larger, the vulnerability code in the SARD project is a fragment of code samples constructed artificially by imitating the vulnerability pattern, and its vulnerability characteristics are significant and can be characterized intuitively from the semantic metric, function granularity, and line-granularity code metric, so the detection results for CWE-399 are the best in these three data sets. In Figure 3, the distribution of CWE-119 samples has a smaller space, and a large number of samples are in the same metric taking range, resulting in the difference between positive and negative samples which is not as obvious as that of CWE-399 vulnerability types, and most of its samples come from NVD real-world open-source software projects, although after processing by techniques such as code slicing and semantic replacement, its vulnerability characteristics are not as significant for the SARD samples. However, synthesizing the data in Table 7, the deviation of the overall vulnerability detection effect is within an acceptable range, and the maximum difference of *F*_1_ measure is 2.7%, which indicates that the SVDM is universally applicable to different vulnerability types.

RETRACTED

To further illustrate the effectiveness of the SVDM, this paper conducts the same training and testing on a unified benchmark for Flawfinder, RIPS, VCCFinder, VPM, and VulExplore, using the same data set as the multiscale code metric data set constructed in Section 2 (Multi-SET), and the detection results are shown in Table 8.

From Table 8, the detection results of the method proposed in this paper are better than other vulnerability detection tools or methods. The SVDM sets corresponding feature extraction layers according to the characteristics of different level code metrics, which makes the vectorized code VCCFinder, VPM, and VulExplore, and all three vulnerability detection methods are based on a single-scale code metric, although in terms of the learning method for code characterization, VCCFinder uses SVM for learning. VCCFinder uses SVM for binary classification, VPM uses Multi-Layer Perceptron (MLP), and VulExplore utilizes CNN + LSTM learning model; each of these methods differs, but the amount of semantic information contained in single-scale code metrics cannot be compared with multiscale code metrics. Flawfinder and RIPS vulnerability detection mainly rely on expert-defined feature rules, when the vulnerability features are not within the defined scope, or the code is very similar to the defined features that will be missed and false positives, which is also the reason for the relatively low detection results. This is the fundamental reason for the gap between traditional tools and deep learning-based methods. For completeness, the Receiver Operating Characteristic (ROC) curves for different tools and methods are shown in Figure 6.

RETRACTED

As shown in Figure 6(a), the ROC curve of the SFN vulnerability detection model tends to be closer to the upper left top. Compared with other tools and methods, SVDM utilizes the Bi-LSTM + CNN + CNN structure for feature extraction and then uses the excellent long-term memory capability of the Bi-LSTM network for deep representation learning, which preserves and incorporates the features of the vulnerable code at different granularities while avoiding gradient disappearance and gradient explosion.  Figure 6(b) shows that the ROC curve of the SFN vulnerability detection model is due to CNN + LSTM, DNN, and LSTM networks. This is because SFN focuses on code context semantic information while also focusing on correlations between metric attributes rather than discrete features. The complementarity of semantic and external features of the code cannot be achieved by a single network, which explains why the SVDM has better performance.

In order to more comprehensively demonstrate the effectiveness and superiority of the method, modifications were made to some parts of the network structures based on the existing model, including the network structure of the SFN and the network structure of the representation learning module. Tables 9 and 10 show the differences between the different models and the detection results of the above models on the unified multiscale code metric data set, respectively.

As shown in Table 9, except for the SVDM, the other four models are all variants of this model.  Table 10 shows the detection results of these five models. First, for the SFN(CNN) + Bi-LSTM, which replaces the Bi-LSTM layer in the feature extraction module, the detection metrics are lower than those of the proposed vulnerability detection model. The reason for this is that the semantic metric part of the multiscale code metric data set is based on the code slicing of contextual semantic relations, and the LSTM neurons in Bi-LSTM are much better than the CNN model in contextual prediction, which is why the temporal network model is chosen in natural language processing. The Bi-LSTM + Bi-LSTM replaces the entire feature extraction module with a Bi-LSTM network, which cannot better define the relationship between metric attributes for code features with strong discrete relationships between attributes and weak temporal sequencings like function and line-level code metrics, which has similar reasons to the SFN (CNN) + Bi-LSTM model in this regard. The DNN module in the SFN+DNN model and the SVM module in the SFN+SVM model given in Table 9, respectively, replace the representation learning model in the proposed SVDM. Bi-LSTM networks of learning modules are replaced with DNN and SVM. For the model replaced with DNN, although its network structure is deep and complex, the information processing in a single neuron is simply linear from input to output, which can be expressed as in the following formula:

(1) $$\begin{array}{c} S_{\text{output}}=\sum_{i=1}^{m}\omega_{i}x_{i}+b. \end{array}$$

When the DNN faces complex nonlinear vectors, as the neural network deepens, the optimization function is getting stuck in a local optimal solution, which leads to results deviating increasingly from the global optimal solution; at the same time, depending on the activation function, the problem of gradient disappearance or gradient explosion easily occurs, for example, when choosing sigmoid as the activation function of neurons, backpropagation of one layer will lead to gradient decay of 0.25, resulting in the underlying neurons not receiving an effective training signal; thus, the detection of SFN + DNN is performed inefficiently. For SFN + SVM, the Bi-LSTM network is replaced by the classical algorithm of machine learning, SVM, similar to DNN that has better results for this linear structure, but for the output of the complex vector by the feature extraction module, SVM cannot be better handled, resulting in significantly lower detection results for each index than other deep learning-based vulnerability detection models.

RETRACTED

Finally, in order to verify how different levels of code metrics would affect the effectiveness of SVDM, this paper adopts the control variable method to combine three different granularity of code metrics in the multiscale code metrics data set and adjust the network structure of the SFN feature extraction model correspondingly for the experiments. The details and structure of the data set and feature extraction model used in this experiment are shown in Table 11.

In Table 11, the datasets utilized for Type-1 through Type-7 are subsets of Multi-SET, which are constructed by manipulating the combination of code metrics at different granularities.

As can be seen in Table 12, the Type-7 control group has the best detection results among all experimental groups. First, in Type-1 and Type-2 experiments, the data sets consist of line-level code metrics and function-level code metrics, respectively, while the traditional code metrics based on text features and code complexity obtain the corresponding code representation sequences through several metrics, which are suitable for quantitative statistical analysis and have faster detection speed, but because the code metrics are based on the overall properties of the program, they do not have a strong correlation with the vulnerability code itself, resulting in poor detection results. Type-3 experiments use token-based semantic metrics to characterize the source code, which has richer source code semantic information than the traditional code metrics. The token sequences obtained directly from the code level statistics have a stronger correlation with vulnerabilities, and the vulnerability patterns contained in them are more clearly expressed in the vector space, so the detection results are better. Similar to Type-1 and Type-2, the data used in Type-4 experiments are a combination of line and function-level code metrics, which is similar to the VulExplore vulnerability detection model proposed by the authors in their previous study. However, in the representation learning phase, Bi-LSTM is less sensitive to the traditional code metrics which are discrete and do not contain contextual semantic information and cannot effectively exploit the advantages of Bi-LSTM. Even though the detection results are higher than the evaluation metrics of Type-1 and Type-2 experiment types, they still have a certain gap compared to the semantic metrics which contain rich contextual semantic information. The data sets in Type-5 and Type-6 experiments are a combination of semantic metrics and two traditional code metrics, respectively. This combination adds the text and complexity measures to the semantic metrics and characterizes a piece of code from a more comprehensive perspective, not only considering the contextual semantic information of the source code, but its overall program-based properties complement the characterization approach from the side. Therefore, Type-7 experiments, i.e., the proposed SVDM, have the best detection results on the multiscale code metric data set with a significant improvement compared to other combinations of code metrics.

RETRACTED

## 4. Related Work

Researchers have proposed many approaches to source-code-oriented vulnerability detection. According to the detection approach, we classify previous research into three types: rule-based, similarity-based, and pattern-based methods.

### 4.1. Rule-Based

The process of detection relies heavily on rules defined by human experts in rule-based vulnerability detection. Some previous tools described vulnerabilities with the help of simple rules and matched the software to be detected with these rules, such as open-source software like Flawfinder [11], Cvechecker [12], and Splint [13]. Some commercial software such as Checkmarx [14] and Coverity [15] also leverage predefined detection rules. In addition, researchers have worked a lot on vulnerability rules, but these studies usually address some aspects of the rules.

### 4.2. Similarity-Based

Due to the prevalence of open source, vulnerabilities caused by code cloning are widely available. Generally, when a piece of open-source code with vulnerabilities is cloned, the vulnerability is also propagated. Similarity-based vulnerability detection determines the similarity between the code and the template with the help of intermediate representations, such as tokens and graphs, to achieve the purpose of vulnerability detection.

To address software security problems caused by code cloning, VulPecker [16] characterizes patches by defining a set of features and proposes a code similarity detection algorithm for different software projects to detect code containing the same vulnerabilities in different projects. The experimental results showed that VulPecker detected 40 vulnerabilities that were not published. Jang et al. proposed the ReDeBug [17] detection method with code behavior granularity using a sliding window approach in the source code and a Bloom filter between files for vulnerability code clone detection. However, ReDeBug only targets code clones of the type of adding, deleting, or modifying statements, resulting in numbers of vulnerable code clones being missed. In addition, the lack of contextual semantic information about the vulnerable code is not taken into account because the approach only uses line-level granularity, which leads to an increase in false positives for detection. To address the current situation where existing work requires a large amount of labeled data, Sun et al. prepared a smaller data set consisting of vulnerabilities and associated patches and attempted to detect similarity in terms of similarity between vulnerabilities and differences between a pair of vulnerabilities and patches. To this end, they constructed VDSimilar [18], a joint detection model using Siamese networks, Bi-LSTM, and Attention to process source code. The proposed model achieves an AUC value of 97.17 on OpenSSL and Linux on a data set of 876 samples. To address the problems of high false positives and poor performance when analyzing large programs, Cui et al. propose to use the weighted feature graph (WFG), a small but semantically rich graph to characterize functions and build a static VulDetector [19]. VulDetector firstly seeks vulnerability-sensitive keywords to reduce the size of the graph without compromising security-related semantics. Then, WFG is used to characterize the code slices and exploit the correlation between vulnerability graphs and patch graphs to improve the accuracy of vulnerability detection. Experiments show that VulDetector achieves an *F*_1_ value of over 81% and detects three vulnerabilities in a real-world project (OpenSSL).

RETRACTED

### 4.3. Pattern-Based

Pattern-based approaches aim to determine whether a target code is vulnerable by learning vulnerability patterns consciously through neural networks. At this stage, these studies free up the workload of human experts in the task of defining vulnerabilities.

VulDeePecker [20] is the first approach to utilize deep learning in vulnerability detection. Li et al. process code slices as Code gadget and then transformed the Code gadget into a vector that can be received by the neural network through word embedding, which is used to train a Bi-LSTM for vulnerability detection, thus proposing the VulDeePecker vulnerability detection system. This method achieves a lower false-negative rate than other vulnerability detection methods; applying VulDeePecker to three software products (Xen, Seamonkey, and Libav), four never-reported vulnerabilities were detected. An et al. proposed an automatic vulnerability detection framework (HAN) [21] based on hierarchical representation and attention mechanism, in which the framework uses five different granularity code slices according to the semantics of the source code during source code representation instead of functions, files, or components to increase the engineering structure information, which can better characterize vulnerabilities and improve detection accuracy; in addition, a hierarchical attention mechanism is added to the HAN framework to highlight the parts that have the greatest impact on classification decisions. Experimental results show that the framework achieves better results in terms of precision and recall metrics.

Code metrics, as a set of sequences characterizing source code, also possess better results in vulnerability detection. In recent years, the increasing degree of open source, the increasing size of software pages, and the lack of expertise of many developers due to the lowered threshold of software development have led to the fact that not all codes are adequately audited. Given the high cost of code auditing through manual work, Perl et al. propose a new approach to find potential vulnerabilities in the code base, VCCFinder [22], by mapping code metrics to the original code and training an SVM classifier to flag flawed code. Compared to the traditional code metric analysis tool Flawfinder, VCCFinder reduces the false-positive rate by 99% for the same recall benchmark. Zagane et al. [23] constructed a data set containing 16 code metrics from publicly available data sets and, unlike previous approaches using long- and short-term memory networks and K-neighborhood algorithms, the proposed vulnerability detection model uses Multi-Layer Perceptron (MLP) for representation learning and achieves 76.9% accuracy in the real-world code metric data set. In addition, based on the existing code metric-based vulnerability detection, Guo et al. [24] constructed a data set containing 21 code metrics, including two new complexity metrics, and proposed a compound deep learning-based vulnerability model VulExplore for this data set. The model obtained a precision of over 81% and reduced both the FNR and FPR to under 20%.

RETRACTED

## 5. Conclusion

In this paper, we first analyze and describe the research background and current status of vulnerability detection and point out the current shortcomings and defects. The current vulnerability detection technology mainly relies on expert experience and rule features, and automated detection has a high FNR and FPR, making it difficult to carry out effective applications. Some new vulnerability detection algorithms have shortcomings in their research results, such as feature extraction is not deep enough to characterize the source code, the network model is prone to overfitting, and the algorithm training costs are high. To solve these problems, the SFN based on Continuous Bag of Words and Convolutional Neural Networks is proposed. The experimental results show that the proposed SFN can effectively improve the performance of feature extraction, and the SVDM vulnerability detection model constructed by SFN and Bi-LSTM also shows better detection results, improving the precision, recall, and F1 while reducing the FNR and FPR.

The effectiveness of multiscale code metrics and SFN for vulnerability detection has been demonstrated, but the current study also has the following limitations:

1. At present, the multiscale code metrics constructed in this paper only cover semantic metrics, function granularity metrics, and line granularity metrics, which are not comprehensive enough for source code. It is a challenging task to find a more complete way to characterize source code.
2. The sources of the multiscale code metric data set constructed in this paper are mainly CWE-119 and CWE-399. Although the predictions for multitype vulnerability detection are also made in the paper, the actual results are not yet known. In addition, the source code detection of multiple vulnerabilities will continue to be studied in future work.
3. The vulnerability detection model proposed in this paper is currently only oriented to programs written in C/C++. Although the detection method of the model is generalizable, the functional modules need to be modified accordingly.

## Figures and Tables

**Figure 1:** The code slice for function-code metric extraction.

**Figure 2:** The code slice for line-code metric extraction.

RETRACTED

**Figure 3:** The architecture of SFN.

**Figure 4:** CWE-119 sample space of distribution.

**Figure 5:** CWE-399 sample space of distribution.

**Figure 6:** (a) The ROC curves of different vulnerability detection methods. (b) The ROC curves of different network models. The closer the curve is to the upper left corner of the graph, the result of the detection is better.

**Table 1:** Function granularity metrics.

Function granularity metrics	Formulas
Program length (*N*)	*N*=*N*_1_+*N*_2_
Number of delivered bugs (*B*)	*B*=(*V*/3000)
Difficulty (*D*)	*D*=(*η*_1_/2)*∗*(*N*_2_/*η*_2_)
Effort (*E*)	*E*=*D∗V*
Time required to program (*T*)	*T*=(*E*/18)
Volume (*V*)	*V*=*N∗* log_2_ *η*
Calculated program length ($\hat{N}$)	$\hat{N}=\eta_{1}{\text{log}}_{2}\eta_{1}+\eta_{2}{\text{log}}_{2}\eta_{2}$
McCabe number (CC)	CC=*e* − *n*+2*p*
Maintainability (*M*)	*M*=max(0, (171 − 5.2*∗*In(*V*) − 0.23*∗*CC − 16.2*∗*In(LOC))*∗*(100/171))
The number of committed bugs per line (*O*)	*O*=(*N*/LOC)*∗*(1/*B*)

*Note*: *N*_1_, *N*_2_ are the total number of all operators and the total number of operands in this sample, *η*_1_, *η*_2_ are the number of different operators and the number of different operands, respectively. In this subsection, we give a code slice as a sample of functional granularity code metric extraction. This code slice is from constructed from CWE-119-CVE-2010-1444-vlc_media_player_1.1.0_CVE-2010-1444_zipstream.c as shown in Figure 1.

**Table 2:** The calculation results of function granularity metrics.

Function granularity metrics	Calculation results
Program length (*N*)	*N*=46
Number of delivered bugs (*B*)	*B*=0.000333
Difficulty (*D*)	*D*=3
Effort (*E*)	*E*=606.139804
Time required to program (*T*)	*T*=33.674434
Volume (*V*)	*V*=202.046601
Calculated program length ($\hat{N}$)	$\hat{N}=72.954453$
McCab number (CC)	CC=2
Maintainability (*M*)	*M*=52.883185
The number of committed bugs per line (*O*)	*O*=0.0030636

**Table 3:** The calculation results of line granularity metrics.

Line granularity metrics	Calculation results
Empty lines	0
Lines of comments	0
Lines of codes (LOC)	5
Physic lines (PLOC)	5
Number of distinct operators (*η*_1_)	7
Number of distinct operands (*η*_2_)	14
Program vocabulary (*η*)	21
Total number of operators (*N*_1_)	26
Total number of operands (*N*_2_)	20

**Table 4:** Software and hardware configuration of the experiment.

Hardware	CPU	Intel I9-10900K
	GPU	NVIDIA GeForce GTX 2080Ti 11G *∗* 2
	RAM	64 GB
	Hard disc	500G M.2 SSD

Software	Operation system	Ubuntu 20.04.3 server
	*Python*	3.7.6
	Keras	2.3.1

**Table 5:** Evaluation indicators.

Indicators	Formulas
Precision	*P*=((TP)/(TP+FP))
Recall	*R*=(TP)/(TP+FN)
FNR	FNR=(FN)/(FN+TP)
FPR	FPR=(FP)/(FP+TN)
*F*_1_	*F*_1_=(2*∗*Precision*∗*Recall)/(Precision+Recall)

RETRACTED

**Table 6:** Experimental results of sampling.

Data set	*P* (%)	*R* (%)	FNR (%)	FPR (%)	*F*_1_ (%)
Sampled	84.3	83.4	16.6	15.7	84.1
Unsampled	80.5	85.8	82.4	85.6	79.8

**Table 7:** Experiment indicators comparison for different data sets.

Data set	Precision (%)	Recall (%)	FN (%)	FP (%)	*F*_1_ (%)
CWE-119-SET	82.6	82.2	17.8	17.3	82.4
CWE-399-SET	**85.2**	**84.8**	**15.2**	**14.7**	**85.1**
Multi-SET	84.3	83.4	16.6	15.7	84.1

**Table 8:** Detection results of different tools or methods.

Methods	Precision (%)	Recall (%)	FN (%)	FP (%)	*F*_1_ (%)
Flawfinder	25.0	31.0	69.0	44.7	27.7
RIPS	48.7	39.5	60.4	51.3	44.5
VCCFinder	57.6	34.1	65.2	43.8	49.2
VPM	74.3	75.9	24.2	26.4	75.3
VulExplore	80.1	81.9	18.8	19.6	81.2
SVDM	**84.3**	**83.4**	**16.6**	**15.7**	**84.1**

**Table 9:** Differences between proposed methods.

Methods	Distinction
SFN + Bi-LSTM	The proposed method
SFN(CNN) + Bi-LSTM	In the SFN feature extraction module, all feature extraction layers are replaced by CNN
Bi-LSTM + Bi-LSTM	SFN feature extraction module replaced with Bi-LSTM network
SFN + DNN	The Bi-LSTM is replaced with a fully connected network in the representation learning module
SFN + SVM	The Bi-LSTM is replaced with a Multi-Layer Perceptron in the representation learning module

**Table 10:** Experimental results of proposed methods.

Methods	*P* (%)	*R* (%)	FNR (%)	FPR (%)	*F*_1_ (%)
SVDM	**84.3**	**83.4**	**16.6**	**15.9**	**84.1**
SFN(CNN) + Bi-LSTM	82.1	81.5	18.4	18.3	81.6
Bi-LSTM + Bi-LSTM	82.9	82.5	17.5	18.6	82.7
SFN + DNN	81.6	80.9	19.1	20.2	81.4
SFN + SVM	73.8	72.2	27.8	27.8	72.7

**Table 11:** Control variable experiment and feature extraction model structure.

Type	Metric granularity	Feature extraction model structure
Type-1	Line	CNN
Type-2	Function	CNN
Type-3	Semantic	Bi-LSTM
Type-4	Line + function	CNN + CNN
Type-5	Semantic + line	Bi-LSTM + CNN
Type-6	Semantic + function	Bi-LSTM + CNN
Type-7	Semantic + line + function	Bi-LSTM + CNN + CNN

**Table 12:** Experimental results of the controlled variable method.

Methods	*P* (%)	*R* (%)	FNR (%)	FPR (%)	*F*_1_ (%)
Type-1	72.9	70.4	29.6	27.1	71.7
Type-2	74.5	71.3	28.7	25.6	72.8
Type-3	80.6	81.2	17.82	18.3	80.9
Type-4	78.2	76.9	23.1	21.7	77.4
Type-5	82.4	82.9	17.1	17.5	82.6
Type-6	83.7	83.1	16.9	16.2	83.4
Type-7	**84.3**	**83.4**	**16.6**	**15.7**	**84.1**

## Data Availability

No data were used to support this study.
